# The lncRNA Signatures of Genome Instability to Predict Survival in Patients with Renal Cancer

This article has been retracted.

**DOI:** 10.1155/2021/1090698

**Published:** 2021-12-07

**Authors:** Liang Huang, Yu Xie, Shusuan Jiang, Weiqing Han, Fanchang Zeng, Daoyuan Li

**Affiliations:** ^1^Department of Urology, The Affiliated Cancer Hospital of Xiangya School of Medicine, Central South University, Hunan Cancer Hospital, Changsha, Hunan 410013, China; ^2^Department of Urology, Hainan General Hospital (Hainan Affiliated Hospital of Hainan Medical University), Haikou, Hainan 570311, China

## Abstract

Long noncoding RNAs (lncRNAs) exert an increasingly important effect on genome instability and the prognosis of cancer patients. The present research established a computational framework originating from the mutation assumption combining lncRNA expression profile and somatic mutation profile in the genome of renal cancer to assess the effect of lncRNAs on the gene instability of renal cancer. A total of 45 differentially expressed lncRNAs were evaluated to be genome-instability-associated from the high and low cumulative somatic mutations groups. Then we established a prognosis model based on three genome-instability-associated lncRNAs (AC156455.1, AC016405.3, and LINC01234)-GlncScore. The GlncScore was then verified in testing cohort and the total TCGA renal cancer cohort. The GlncScore was evaluated to have an accurate prediction for the survival of patients. Furthermore, GlncScore was associated with somatic mutation patterns, indicating its capacity of reflecting genome instability in renal cancer. In conclusion, this study evaluated the effect of lncRNAs on genome instability of renal cancer and provided new hidden cancer biomarkers related to genome instability in renal cancer.

## 1. Introduction

Renal cancer (RC) occupies approximately 3% of all adult malignancies as the twelfth most common cancer across the world [1, 2]. Nephrectomy is the only radical treatment for localized RC [3]. However, 30% of patients were evaluated to have local tumor recurrence or distant metastasis when diagnosed [4]. Metastatic renal cell carcinoma with poor prognosis is not sensitive to radiotherapy and chemotherapy, and the 5-year overall survival is less than 10%. Recently, gene therapy and antitumor angiogenesis molecular targeted drugs significantly improved the prognosis of the RC [5]. However, due to the complexity of biological behavior of renal cell carcinoma, there is a lack of effective molecular markers to predict the prognosis and treatment response of renal cell carcinoma [6, 7].

Long noncoding RNAs (lncRNAs) have been great players in almost every extent of gene function and control [8]. Recently, lncRNAs were evaluated to exert a significant effect on keeping genome instability [9]. With the maturity and application of high-throughput detection technology and the rapid development of bioinformatics, the expression regulation functions of lncRNA have been discovered one after another, which not only enriches the complexity of the genome but also makes us realize some abnormalities of lncRNA in renal cancer. The expression situation makes our research on the link between lncRNA and kidney cancer more in-depth. However, the biological understanding of lncRNA in renal cell carcinoma is still slow, and its function and mechanism are still unclear. Moreover, there are few lncRNAs closely related to renal cell carcinoma.

As we have known, the genome instability is not only a marker of cancer but also an important prognostic factor because it is related to tumor progression and survival. lncRNA NORAD has been shown to contribute to genome stability through the ability modulation of an RNA-binding protein for assembling a higher-order ribonucleoprotein complex [10]. It has been shown that several other lncRNAs take part in genome stability [9]. However, there are largely unexplored genome-instability-related lncRNAs and their clinical significance in RC.

## 2. Methods

### 2.1. Data Collection and Recognition of Genome-Instability-Associated lncRNAs

The clinical characteristics, RNA-seq expression information, and somatic mutation data of RC patients were obtained from The Cancer Genome Atlas (TCGA) database. We obtained the mutation frequency of each patient and defined patients with the top 25% highest mutation frequency as the high mutation group (GU group) and patients with the lowest 25% mutation frequency as the low mutation group (GS group). lncRNAs related to genome instability were defined as the differentially expressed lncRNAs (fold variation >1.5 or <0.67 and false discovery rate (FDR) modified *P* < 0.05) between the GU and GS groups.

### 2.2. Functional Improvement Analysis

The relationship between the paired expression of genome-instability-related lncRNAs and mRNAs was measured by computing the Pearson correlation coefficients, and the top 10 mRNAs were regarded as coexpressed genome-instability-related lncRNA-related partners. For predicting the hidden roles of genome-instability-associated lncRNAs, obviously enriched Gene Ontology (GO) terms and Kyoto Encyclopedia of Genes and Genomes (KEGG) pathway were determined by performing functional improvement analysis of coexpressed lncRNA-related mRNA partners. ClusterProfiler package in R software was employed to make the function enrichment analysis.

*The Research on a Genome-Instability-Originated lncRNA Signature for Survival Forecast*. We used the genome-instability-derived lncRNAs to develop a model for survival prediction. The outcome was set as the overall survival which was defined as the survival from date of inclusion until the death of patients. All patients with RC were randomly divided into training group and test group. The training set is mainly adopted for the identification of the prognostic lncRNA and the construction of predictive risk model; the test set is mainly adopted for the verification of the prognostic risk model.

### 2.3. Statistical Analysis

R version 4.0.3 was employed to make all statistical analyses. The correlation between the expression extent of lncRNA related to genomic instability and entire survival was evaluated with univariate and multivariate Cox proportional hazards regression analysis. On the basis of the parameters of multiple regression analysis and the expression extent of lncRNAs related to prognostic genomic instability, genomic-instability-derived lncRNA features (GlncScore) were constructed for result forecast. Taking the median score of the patients in the training set as the critical value of risk, the patients fall into high-risk group with high GlncScore or low-risk group with low GlncScore. The survival rate and median survival rate of every prognostic risk group were calculated with Kaplan-Meier approach, and the diversity in survival rate between the high-risk group and the low-risk group with a significant level of 5% was evaluated with the log-rank test. A time-related receiver operating characteristic curve (ROC) was adopted to assess the performance of GlncScore.

## 3. Results

### 3.1. Recognition of lncRNAs Related to Genome Instability in Renal Cancer

According to the cell mutation of patients with renal clear cell carcinoma from TCGA database, the comparison of expression differences of lncRNAs between GU group and GS group was made in descending order. Finally, 45 lncRNAs were found to have significant differences in expression: 15 upregulated lncRNAs and 30 downregulated lncRNAs in GU group (Figure 1(a) and Supplementary Table 1). A total of 692 patients with renal cancer with complete clinical data were included in the subsequent analysis. The 45 lncRNAs were used to cluster 692 TCGA unsupervised samples.

### 3.2. Identification of Potential Functions

We used gene enrichment analysis to predict the hidden roles of 45 lncRNAs associated with genome instability. By measuring the association between 45 differentially expressed lncRNAs and protein coding genes, we got the top 10 most closely related lncRNAs and mRNAs for the construction of the lncRNA-mRNA coexpression network (Figure 2(a)). Furthermore, GO analysis displayed that the mRNAs in this coexpression network were related to the generation and development of genome instability (Figures 2(b) and 2(c)). According to the analysis of KEGG pathway, there were several pathways that were significantly enriched, including vascular smooth muscle contraction, cell adhesion molecules, and chemokine signaling pathway (Figures 2(d) and 2(e)). According to the above outcomes, the 45 differentially expressed lncRNAs were regarded as candidate lncRNAs related to genome instability.

### 3.3. Establishment of Prognosis Model of Clear Cell Renal Cell Carcinoma

For the further study of the prognostic effect of the above candidate lncRNAs, 692 patients with renal cancer from TCGA database were divided into training group and test group, with 346 patients in training group. The baseline characteristics of the training and test groups were well balanced as shown in Supplementary Table 2. In the training group, the univariate Cox proportional hazards regression analysis was adopted to explore the association between the 45 lncRNAs related to gene instability and overall survival, of which 3 lncRNAs were greatly related to the prognosis of patients (*P* < 0.05; Figure 3(a)). Next, multivariate Cox proportional hazards regression analysis was made among the 3 candidate lncRNAs as well as usual clinical characteristics including age, gender, pathological phase, and TNM phase. Finally, all three candidate lncRNAs (AC156455.1, AC016405.3, and LINC01234) were recognized as independent prognostic lncRNAs as their prognostic significance in multivariate Cox (*P* ＜ 0.05) was retained. Finally, we constructed a genome-instability-originated lncRNAs signature (GlncScore) to evaluate the prognostic risk of patients with renal cancer by combining the correlation coefficient of multivariate Cox analysis and the expression extent of three independent prognostic lncRNAs. The formula of the GlncScore is as follows:

(1) $$\begin{array}{c} \text{GlncScore}=0.823*\text{ expr}\left(\text{AC}156455.1\right)+0.211*\text{ expr}\left(\text{AC}016405.3\right)+0.139*\text{expr}\left(\text{LINC}01234\right). \end{array}$$

On the basis of the median value of risk score, patients fell into high-risk group (the value of risk score is higher than the median value) and low-risk group (the value of risk score is lower than the median value). Kaplan-Meier analysis showed that the survival outcomes of patients in the low-risk group are greatly better than those of patients in the high-risk group (*P* < 0.05, log-rank test; Figure 3(b)). The time-dependent ROC curves analysis of the GlncScore showed an area under curve (AUC) of 0.778 (Figure 3(e)). The patients of the high-risk group had a significantly high level of somatic mutations compared with those of the low-risk group (Figure 4(a)).

### 3.4. Validation of GlncScore

The 346 patients of the testing set were divided into a high-risk group and a low-risk group with greatly varied overall survival. According to Figure 3(c), patients in the high-risk group showed much poorer entire survival than patients in the low-risk group. The time-dependent ROC curves analysis of the GlncScore in the testing set showed an AUC of 0.807 (Figure 3(f)). The allocation of somatic mutation count in the testing samples was illustrated in Figure 4(b). The prognostic performance of the GlncScore in the whole TCGA set was like the above outcomes.

### 3.5. Independence of the GlncScore from Other Clinical Elements

The multivariate Cox regression analyses were made on age, gender, grade, phase, and our GlncScore. The GlncScore was greatly related to overall survival (Table 1). We divided the patients in TCGA database into young group and elderly group based on 60 years of age. The patients in every age group can be further divided into a high-risk group and a low-risk group. A great diversity in the survival rate between the high-risk group and the low-risk group in the young group (log-rank test, *P*=0.012; Figure 5(a)) was observed, which was also applicable to the elderly group (log-rank test, *P*=0.001; Figure 5(b)). Similarly, the patients in TCGA database were divided into male group and female group. Patients of each gender were further divided into a high-risk group and a low-risk group. Great diversities in survival rates among female patients but not among male patients (Figure 5(c) and 5(d)) were observed. Furthermore, we grouped the pathological stages of renal cancer patients in TCGA database; pathological phases I and II were integrated into early group, and pathological phases III and IV were integrated into late group. Then the patients in the early group and the late group were further divided into a high-risk group and a low-risk group. The survival rates of the patients in the early group and the late group were significantly different (Figure 5(e) and F). According to these outcomes, the GlncScore was an independent prognostic element related to entire survival in kidney cancer patients.

## 4. Discussion

In recent years, a number of studies have been carried out on the occurrence, development, and treatment of renal cancer [11, 12]. The incidence of kidney cancer has been on the rise in recent years. The diagnosis and staging of kidney cancer are of great significance to its treatment and prognosis. Multislice spiral CT is of great significance in the diagnosis of kidney cancer and is superior to other examinations. Doppler ultrasonography is difficult to characterize the tissue of renal tumors, and it is easy to miss the diagnosis of small tumors. The application of the new ultrasound contrast agent sonovir in renal tumors is still in the exploratory stage. MRI is difficult to use as a routine examination. Radical nephrectomy is an accepted method for the treatment of locally advanced renal cancer. Minimally invasive treatment such as laparoscopic surgery is the current development trend and is gradually mature. Stem cell transplantation, targeted antigens, and tumor vaccines are currently hot research directions.

Radical nephrectomy is still the most effective treatment for locally advanced renal cancer; and whether it is necessary to perform lymph node dissection, venous tumor thrombus removal, ipsilateral adrenalectomy, and so forth should be based on the corresponding treatment principles and different patients. According to the individual situation, the most suitable surgical treatment plan can be formulated. The choice of incision for kidney surgery is a very important preoperative thinking problem for surgeons. The basic idea should be to quickly and effectively control the renal arteries and veins to ensure the safety of the operation, facilitate the free nephrectomy of kidney tumors, and meet the tumor-free operation of tumor surgery. The first two are the most important starting points for the selection of surgical approaches. For small kidney cancer or kidney cancer that is difficult to operate, kidney-sparing surgery is advocated. The 23rd World Congress of Urology Endoscopy unanimously agreed that nephron-preserving surgery is suitable for kidney cancer with a diameter of ≤4 cm. NSS includes partial nephrectomy (laparoscopic or laparoscopy), tumor rejection, radiofrequency ablation, cryoablation, arterial chemoembolization, laser ablation, and ultrasound energy accumulation. The purpose of minimally invasive treatment is to preserve normal kidney tissue as much as possible and minimize complications.

The incidence of kidney cancer is still increasing by 3% every year in the world. Because there is no early diagnosis and warning method, about half of newly diagnosed patients develop locally advanced kidney cancer or metastatic kidney cancer, while metastatic kidney cancer only takes an average of 10 months as the lifetime. The insensitivity of conventional radiotherapy and chemotherapy to kidney cancer results in the lack of means to prevent the recurrence and metastasis of kidney cancer; it also hinders the realization of the goal of improving the quality of life of advanced kidney cancer and prolonging the survival period of advanced kidney cancer. Sorafenib, a targeted drug for the treatment of advanced renal cell carcinoma, was first approved by the U.S. FDA in 2005, followed by sunitinib, axitinib, pazopanib, temsirolimus, everolimus, and benzalkonium chloride. Varizumab has been approved for the market, opening a new chapter for the treatment of advanced kidney cancer. The key to the treatment of kidney cancer with targeted drugs lies in how to adjust the dose of the drugs and at the same time discovering, reducing, and dealing with the side effects caused by targeted drug treatments, especially in the first month of treatment, are very important. Kidney cancer has a variety of immune correlations, and the clinical efficacy of multiple immunotherapies for renal cancer has been widely used. The immunotherapy of kidney cancer covers immune targeted therapy, combined immune targeted therapy, and immunotherapy combined with immune checkpoint blocking, kidney cancer vaccines, cytokines, and adoptive cells. IL-2 treatment of kidney cancer CAIX has become a screening indicator, which opens up a new direction for selective immunotherapy of kidney cancer. At the same time, in the in-depth study of the interaction of renal cancer immunotherapy, CTLA-4, and immune checkpoint antibody PD-1, new immunotherapeutic factors have brought new hope to clinical immunotherapy of renal cancer. However, the judgment of the efficacy of combined immunotherapy for kidney cancer may be due to the different responses of patients to immunotherapy and individual differences. More evidence-based medicine research is needed. With further research on the molecular level of cancer cells, the development of new vaccines for dendritic cells and tumor antigen preparations will open up new ways for the treatment of patients with advanced renal cancer. In short, it emphasizes regular physical examination, early diagnosis, and early surgical treatment of susceptible people. The diagnosis and treatment of kidney cancer with integrated traditional Chinese and Western medicine are advocated, so Chinese medicine can also play a certain clinical role. The survival rate and quality of life of kidney cancer patients in China will definitely improve.

Individualized treatment of cancer is the trend of cancer treatment [13]. It is very important to predict the possibility of individual recurrence according to prognostic factors for guiding the treatment of patients and individualized monitoring. The genome instability is a common feature of most of the cancers and affects the prognosis of cancer patients [14]. However, the quantitative measurement of genome instability has been a problem faced by many researchers. At the same time, there is evidence that abnormal transcription and epigenetic changes are important factors leading to genome instability.

Recently, increasing attentions have been paid to the role of lncRNAs as cancer biomarkers [15]. Identifying lncRNAs related to genome instability and systematically exploring their clinical significance in RC are still in the infancy period. Although lncRNA lacks the function of encoding protein, its important role in transcriptional regulation is well known, and then it regulates a series of biological processes such as dose compensation, genome imprinting, maintenance of genome integrity, cell cycle control, development, and differentiation [16].

lncRNAs are a class of noncoding RNA molecules with transcripts between 200 nt and 100 kb in length. Most of them are produced by RNA polymerase II transcription. Their subcellular locations are diverse and are distributed in the nucleus, cytoplasm, and organelles. In most of the cases, lncRNAs are longer and have an mRNA-like structure, some have a poly(A) tail, and some do not have a poly(A) tail and have dynamic expression and different splicing methods during the differentiation process. By comparison with the coding gene, the expression level of lncRNA is lower. The expression level of lncRNA between different tissues is not the same, which is not only tissue-specific; at the same time, lncRNA also has temporal and spatial specificity; that is, the expression level of lncRNA in the same tissue or organ at different growth stages can also change. lncRNAs not only exert a significant effect on the pathogenesis of tumors but also exert a great effect on cardiovascular, autoimmune, infectious, and neurological diseases. This study has confirmed that lncRNAs have the following functions: ① Recruiting chromatin remodeling complexes to specific genomic sites and making them catalytically active. ② Transcription of the transcription factor in the upstream promoter area of the protein-encoding gene, involved in the expression of neighboring protein-encoding genes. ③ Inhibiting RNA polymerase II, forming complementary double strands with the transcript of the gene encoding protein, being involved in the shearing of mRNA, and then generating various forms of shearing or generating endogenous sRNA under the action of Dicer enzyme to control gene expression level. ④ Binding to a specific protein regulating the activity of the corresponding protein or changing the cytoplasmic localization of the protein. ⑤ Transcription as the precursor of small molecule RNA, such as miRNAs and piRNA. Abnormal expression of lncRNA can promote the occurrence of many diseases including tumors.

With the maturity and application of high-throughput detection technology and the rapid development of bioinformatics, the expression regulation functions of lncRNAs have been discovered one after another, which not only enriches the complexity of the genome but also makes us realize some abnormalities of lncRNA in renal cancer. The expression situation makes our research on the link between lncRNA and kidney cancer more in-depth. However, the biological understanding of lncRNA in renal cell carcinoma is still slow, and its function and mechanism are still unclear. Moreover, there are few lncRNAs closely related to renal cell carcinoma. In the future, the mechanism of their effect on the occurrence and development of renal cell carcinoma shall be explored further. Existing studies have found the mechanism of abnormal expression of lncRNA in renal cell carcinoma and the mechanism of the influence of abnormal expression of lncRNA on the occurrence, development, metastasis, and invasion of renal cell carcinoma, laying the foundation for our next treatment of renal cell carcinoma. We believe that, with the deepening of research, lncRNAs studies will open a new chapter in the molecular targeted therapy and drug development of renal cancer. lncRNAs can take part in controlling gene expressions at the levels of transcription, posttranscription, and epigenetics, thereby affecting the growth, development, aging, death, and other life processes of the body. Recently, researches have found that lncRNAs have a function similar to oncogenes or tumor suppressor genes and are closely associated with the proliferation, invasion, metastasis, and prognosis of renal cancer cells. This article discusses the research progress of lncRNA in renal cancer and provides a new direction for finding molecular markers and drug targets for renal cancer.

There were several limitations in the current research. First, the GlncScore is on the basis of the computational framework; further experimental research would be needed to understand its regulatory mechanism. Second, the GlncScore should be verified externally to ensure the practicability and repeatability of the model. Third, the influence of different treatment approaches on the predictive accuracy of the model was not evaluated; the future study should perform subgroup analysis based on the treatment the patients received.

## 5. Conclusion

This study identified the lncRNA features derived from genomic instability as an independent prognostic marker for stratifying the risk subgroups of renal cancer patients. Through further prospective verification, GlncScore may be of great significance to the genomic instability and customized decision-making of renal cancer patients [17–20].

## Figures and Tables

**Figure 1:** Recognition of genome-instability-associated lncRNAs among patients suffering from renal cancer. (a) The heatmap of the differentially expressed lncRNAs between GU and GS groups. (b) Unmonitored clustering of 692 renal cancer patients on the basis of the expression pattern of 45 candidate genome-instability-associated lncRNAs. (c) Boxplots of somatic mutations in the GU-like group and GS-like group. (d) Boxplots of UBQLN4 expression level in the GU-like group and GS-like group.

**Figure 2:** The functional concepts of genome-instability-associated lncRNAs in patients with renal cancer. (a) Coexpression network of genome-instability-associated lncRNAs and mRNAs on the basis of the Pearson association parameter. ((b) and (c)) GO analysis for mRNAs coexpressed with lncRNAs. ((d) and (e)) KEGG analysis for mRNAs coexpressed with lncRNAs.

**Figure 3:** Recognition and verification of the genome-instability-derived lncRNA signature (GlncScore) for overall survival forecast. (a) Univariate Cox regression analysis genome-instability-associated lncRNAs related to entire survival in renal cancer. The Kaplan-Meier estimates of entire survival of patients with low or high risk forecast by the GlncScore in the (b) training set, (c) test set, and (d) the whole TCGA renal cancer set. Time-dependent ROC curves analysis of the GlncScore at 3 years in the (e) training set, (f) test set, and (g) the whole TCGA renal cancer set.

**Figure 4:** Distribution of somatic cumulative mutations in the high- and low-risk groups in the (a) training set, (b) test set, and (c) the whole TCGA renal cancer set.

**Figure 5:** The Kaplan-Meier estimates of entire survival of patients with low or high risk forecast by the GlncScore in the (a) young group (≤60 years of age), (b) elderly group (>60 years of age), (c) male group, (d) female group, (e) stages I-II group, and (g) stages III-IV group.

**Table 1:** Multivariate Cox regression analysis of the GlncScore and entire survival in TCGA datasets.

Variables	HR	95% CI	*P* value
GlncScore	1.86	1.23–2.69	0.001
Age	1.94	0.88–4.29	0.098
Gender	1.18	0.37–3.78	0.774
Pathological stage	8.32	2.20–31.34	0.001
Tumor grade	2.23	0.82–6.07	0.113

## Data Availability

The simulation experiment data used to support the findings of this study are available from the corresponding author upon request.

## Supplementary Materials

Supplementary Materials Supplementary Table 1: 45 lncRNAs were found to have significant differences in expression in GU group. Supplementary Table 2: the baseline features of the training and test groups.
